The article "Dicer promotes tumorigenesis by translocating to nucleus to promote SFRP1 promoter methylation in cholangiocarcinoma cells" was published in 2017. Journal: Cell Death Dis.

# Dicer promotes tumorigenesis by translocating to nucleus to promote SFRP1 promoter methylation in cholangiocarcinoma cells

**DOI:** 10.1038/cddis.2017.57

**Published:** 2017-02-23

**Authors:** Wenlong Cheng, Yongqiang Qi, Li Tian, Bing Wang, Wenhua Huang, Yongjun Chen

**Affiliations:** 1 Department of Biliary-Pancreatic Surgery, Tongji Hospital, Tongji Medical College, Huazhong University of Science and Technology, Wuhan, Hubei, China; 2 Department of Vascular Surgery, Wuxi People's Hospital, Nanjing Medical University, Wuxi, Jiangsu, China

## Abstract

Dicer, a member of the RNase III family of endoribonucleases, has an important role in regulating methylation of CpG islands in mammal cancer cells. However, the underlying mechanism of action remains unclear. In this study, we demonstrated that upregulation of Dicer in cholangiocarcinoma (CCA) cells and its translocation to nuclues to interact with heterochromatin protein 1*α* (HP1*α*). The nuclear Dicer/HP1*α* complex appeared to promote both H3K9 trimethylation and DNA methylation of the secreted frizzled-related protein 1 (SFRP1) promoter. The expression of Dicer negatively correlated with that of SFRP1 and it appeared to promote CCA cell proliferation and invasion through repression of *SFRP1* gene. High expression of Dicer in tumor tissues was significantly associated with larger tumor size (>3 cm) and lymph node metastasis. Our findings help characterize the role of Dicer in epigenetic regulation and tumorigenesis in the context of CCA.

Cholangiocarcinoma (CCA), an epithelial cancer of the biliary tract, accounts for 3% of all gastrointestinal tract cancers.^1, 2^ The tumor has a tendency for aggressive growth, is typically difficult to diagnose at an early stage, and is usually fatal because of its late clinical presentation. Most CCAs are unresectable because of early metastasis, and 5-year survival rates are <5%.^3, 4^ Therefore, understanding the molecular pathogenesis of CCA is of much clinical relevance.

Recent studies have underlined the important role of epigenetic aberrations in carcinogenesis and cancer progression. DNA methylation is a widely-studied epigenetic mechanism. Aberrant DNA methylation is an early and stable event in carcinogenesis. Identification of specific DNA methylation patterns may potentially serve as diagnostic markers for early detection and for development of therapeutic modalities.^5^ Genome-wide hypomethylation and specific CpG islands hypermethylation are the most common changes in molecular biology associated with tumors.^6^

Dicer is widely conserved across eukaryotic lineages. It is a member of the RNase III family of endoribonucleases and targets precursor miRNA (pre-miRNA) or long double-stranded RNA (dsRNA) to produce miRNA or siRNA as part of its essential role in various RNA interference (RNAi) pathways.^7, 8^ Dicer is known to regulate methylation of CpG island in mammalian cancer cells;^9, 10, 11, 12^ however, the underlying mechanisms of the same are not clear. In this study, we documented upregulation of Dicer in CCA cells and showed that it translocates to nucleus and interacts with heterochromatin protein 1*α* (HP1*α*). The Dicer/HP1*α* complex promotes DNA methylation of genes which results in repression of transcription. We demonstrate that Dicer promotes CCA cell proliferation and invasion, at least in part, through repression of the secreted frizzled-related protein 1 (*SFRP1*) gene. These results indicate a role of Dicer in epigenetic regulation and tumorigenesis in the context of CCA.

The article "Dicer promotes tumorigenesis by translocating to nucleus to promote SFRP1 promoter methylation in cholangiocarcinoma cells" was published in 2017. Journal: Cell Death Dis.

## Results

### Dicer is upregulated and translocates to nucleus to form complex with HP1*α* in CCA cells

Immunohistochemistry (IHC) staining for Dicer expression was performed in 40 CCA specimens and 13 specimens of anatomically contiguous normal tissues. No significant difference of Dicer expression in the cytoplasm was observed between CCA tissues and peritumoral tissues (mean stain index: non-cancer=4.22±0.58; cancer=5.10±0.66). However, nuclear expression of Dicer in CCA tissues was significantly higher than that in the peritumoral tissues (mean stain index: non-cancer=1.66±0.36; cancer=7.12±0.84) (Figure 1a).

Cytoplasmic and nuclear extracts were then subjected to western blotting to compare the expression of Dicer in CCA cell lines (Hucct1 and TFK1) with that in normal cholangiocyte cell line HIBEpic. The results showed that the Dicer of HIBEpic was mainly located in the cytoplasm. However, its expression in CCA cells was upregulated and most of it translocated to nucleus to play a specific role (Figure 1b).

Considering that Dicer is required for the heterochromatin formation,^13^ and HP1*α* is the symbol protein of the heterochromatin which binds to the domain of trimethylation at Lys9 of histone H3 (H3K9me3), we performed GST pull-down assays to assess any direct interaction between Dicer and HP1*α* in the presence of RNAse. On western blotting, endogenous Dicer (or HP1*α*) proteins from HEK293 cells were captured specifically by GST-HP1*α* (or GST-Dicer), which demonstrated a physical binding of Dicer with HP1*α*, which was independent of RNA *in vitro* (Figure 1c). To further investigate the interplay of these two proteins, we performed co-immunoprecipitation (Co-IP) with nuclear extracts, which revealed an interaction between Dicer and HP1*α* in Hucct1 cells. This interaction was not observable in the HIBEpic cells which had a low nuclear expression of Dicer (Figure 1d). The histone methyltransferase SUV39H1 and DNA methyltransferases (Dnmts) play an important role in epigenetics.^14^ The model of HP1*α*/H3K9me3/SUV39H1/Dnmts complex has been confirmed in several organisms such as Drosophila, mouse and humans.^15, 16^ As shown in Figure 1e, the Co-IP results also verified the model in Hucct1 cells. Collectively, these findings strongly support the hypothesis that Dicer translocates to nucleus and interacts with HP1*α*/H3K9me3/SUV39H1/Dnmts complex in CCA cells.

The article "Dicer promotes tumorigenesis by translocating to nucleus to promote SFRP1 promoter methylation in cholangiocarcinoma cells" was published in 2017. Journal: Cell Death Dis.

### Dicer regulates chromatin modifications in CCA cells

To investigate the role of Dicer in chromatin modifications, we stably silenced Dicer expression through lentiviral-mediated transfection carrying siRNA targeting Dicer in CCA cells (LV-siR-Dicer), and upregulated Dicer expression in HIBEpic cells (as control) through lentiviral-mediated transfection carrying small activating RNA (saRNA) targeting Dicer (LV-saR-Dicer). qRT-PCR and western blot analyses revealed downregulation of Dicer in the LV-siR-Dicer CCA cells (Figures 2a–c). We found upregulation of cytoplasmic expression of Dicer in LV-saR-Dicer HIBEpic cells, but not in the nucleus (Figures 2b and c), which implies that excess Dicer did not translocate from cytoplasm to nucleus. Subsequently, we found lower protein levels of H3K9me3 in LV-siR-Dicer cell lines as compared with that in controls, while the level of H3K9me3 in the LV-saR-Dicer HIBEpic cells showed no change (Figure 2d). In addition, we analyzed the global CpG methylation in Hucct1 cells using a Human Methylation 450 K microarray. A total of 2185 genomic regions (1516 genes) showed significant differences in methylation patterns between LV-siR-Dicer and LV-NC, which included 1055 hypermethylated sites (694 genes) and 1130 hypomethylated sites (822 genes) (Figure 2e). Taken together, Dicer could promote trimethylation of H3K9 and influence genomic methylation patterns in CCA cells.

### Dicer promotes SFRP1 promoter methylation in CCA cells

We next selected eight of the most differentially methylated genes between the LV-siR-Dicer and LV-NC Hucct1 cells, which included four hypermethylated genes and four hypomethylated genes (Figure 3a). Amongst these, *SFRP1*, an antiproliferative tumor suppressor gene located at 8p11.2, is inactivated because of aberrant promoter hypermethylation observed in numerous cancers, such as colorectal cancer^17^ and ovarian cancers.^18^ We investigated whether Dicer could regulate the chromatin modifications of SFRP1 promoter. We researched the CpG islands (CpGs) of SFRP1 promoter and designed primers for ChIP and BSP assays (Figure 3b). ChIP analysis demonstrated reduced Dicer, HP1*α* and H3K9me3 binding in the promoter region of SFRP1 in the LV-siR-Dicer CCA cells as compared with that in the control cells (Figure 3c). Interestingly, upregulation of Dicer in HIBEpic cells had no significant impact on the enrichment of these three proteins to the promoter of SFRP1. Actin promoter control qPCR showed that alterarion of Dicer expression had no significant difference in the enrichment of these three proteins. This proved that the reduction of binding efficiency was not due to global downregulation mechanism, but rather an event specific to some promoter loci. On BSP analysis, CpG methylation of the SFRP1 promoter in LV-siR-Dicer CCA cells was significantly lower than that in the controls (Figure 3d). However, both upregulation and downregulation of Dicer in HIBEpic cells did not significantly impact CpG methylation of the SFRP1 promoter. Collectively, these data suggest that Dicer can promote both H3K9 trimethylation and DNA methylation of SFRP1 in CCA cells through the Dicer/HP1*α*/H3K9me3/SUV39H1/Dnmts complex.

The article "Dicer promotes tumorigenesis by translocating to nucleus to promote SFRP1 promoter methylation in cholangiocarcinoma cells" was published in 2017. Journal: Cell Death Dis.

### Negative correlation between expression of Dicer and SFRP1 in CCA specimens

To verify whether CpG methylation has any regulatory effect on SFRP1 expression in CCA cells, we performed qRT-PCR assays to compare SFRP1 levels in 5-aza-2'-deoxycytidine (5-aza-dC, a DNA methyltransferase inhibitor)-treated and -untreated CCA cells. As shown in Figure 3e, treatment with 5-aza-dC appeared to reverse the expression of SFRP1 in LV-NC CCA cells. The results indicate that expression of SFRP1 was affected by promoter methylation. On western blotting and qRT-PCR assays, downregulation of Dicer was shown to restore expression of SFRP1 because of demethylation (Figures 3f and 4a).

To verify the correlation between Dicer and SFRP1 expression, we tested the mRNA expression of Dicer and SFRP1 in 40 CCA samples. Pearson correlation coefficient of −0.47 (*P*<0.01) indicated a negative correlation between the two (Fig.3 f).

### Dicer promotes proliferation and invasion by silencing SFRP1 expression, inhibits apoptosis of CCA cells and associates with clinicopathology

As stated before, SFRP1 has been shown to be a candidate tumor suppressor gene.^19^ On the basis of our observation that Dicer is functionally involved in promoter methylation and transcriptional silencing of SFRP1 (Figures 3d and 4a), we next investigated a potential role of Dicer in the pathogenesis of CCA. On flow cytometry, the percentage of Hucct1 and TFK1 cells in the S-phase were found to have decreased by 21.36±2.87% and 17.25±1.71%, respectively, as compared with that in the control cells (Figure 4b). Further, downregulation of SFRP1 appeared to partially rescue the percentage of S-phase. Subsequently, we assessed the effects of Dicer on CCA cell proliferation, migration and invasion using CCK-8, wound healing and Transwell assays (Figures 4c–e). Although downregulation of Dicer inhibited cell proliferation and invasion, no significant differences in migration were observed as compared with that in control. Moreover, the downregulated capacity of proliferation and invasion appeared to be partially rescued by transient SFRP1 knockdown. In a study by White *et al.,*^20^ loss of nuclear Dicer resulted in accumulation of dsRNA, which triggered the interferon response pathway, leading to cellular apoptosis. We next detected the protein levels of cleaved caspase-3 and poly ADP-ribose polymerase (PARP) to evaluate apoptosis status after Dicer-silencing. The caspase-3-PARP is a classical apoptosis pathway. The protein expression of cleaved caspase-3 and PARP in the LV-siR-Dicer group was significantly higher than that in the LV-NC group (Figure 4f). However, no significant differences were observed between LV-siR-Dicer and LV-siR-Dicer+siR-SFRP1 groups. The observed phenomenon suggests that downregulation of Dicer led not only to cellular apoptosis in CCA cells but also that the effect was not mediated via the SFRP1 pathway. We finally assessed whether downregulation of Dicer could repress tumor growth *in vivo*. Tumor growth in nude mice from LV-siR-Dicer group was significantly reduced as compared with that in the LV-NC group (Figure 4g). The expression of Dicer and SFRP1 in tumors from nude mice (Figure 4h) was consistent with the functional link between Dicer and SFRP1 described above.

The article "Dicer promotes tumorigenesis by translocating to nucleus to promote SFRP1 promoter methylation in cholangiocarcinoma cells" was published in 2017. Journal: Cell Death Dis.

We then examined the correlation between Dicer expression in the 40 CCA tissue specimens and the clinicopathological. High expression of Dicer in tumor tissues was significantly associated with larger tumor size (>3 cm) and lymph node metastasis, but not with other parameters such as age, sex and pathology grade (Table 1). On cumulative Kaplan–Meier analysis, the 4-year overall survival rate for the 31 patients who had high expression of Dicer (IHC staining index:>6) was significantly lower than that for the nine patients who had low expression of Dicer (IHC staining index:≤6) (Figure 4i).

## Discussion

The results of the present study indicates that Dicer translocates to nucleus and interacts with HP1*α*/H3K9me3/SUV39H1/Dnmts complex for effecting H3K9 trimethylation and DNA methylation at SFRP1 promoter, which results in transcriptional silencing in CCA cells (Figure 5). Thus, Dicer promotes proliferation and invasion of CCA cells, at least in part, through repression of the tumor suppressor SFRP1.

The article "Dicer promotes tumorigenesis by translocating to nucleus to promote SFRP1 promoter methylation in cholangiocarcinoma cells" was published in 2017. Journal: Cell Death Dis.

With the deepening of the research on the structure and function of Dicer, Giles *et al.*^13^ have reported the deficiency of Dicer was shown to cause depolymerization of heterochromatin in vertebrates, which indicates that Dicer is required for heterochromatin formation. In other species, Dicer was demonstrated to link the RNAi pathway with heterochromatin assembly.^20, 21, 22, 23^ Furthermore, Dicer was shown to be indispensable to maintenance of full promoter CpG island hypermethylation in human cancer cells^9^ and in mammalian cells. A reduced Dicer expression was shown to result in a more open chromatin structure due to decreased methylation and increased acetylation of histones. In the present study, we found a similar phenomenon in that the downregulation of Dicer expression reduced H3K9 trimethylation and DNA methylation of target genes such as SFRP1. However, those hypermethylated sites may be attributable to the secondary effects induced by depletion of Dicer (Figure 3a). Interestingly, in a recent article, Gagnon *et al.*^24^ reported co-localization of Dicer, Argonaute-2 (Ago2), TRBP and TRNC6A in human nuclei as part of multi-protein complexes. Some miRNAs are bound to the complexes to complete miRNA pathways. This model inspired us to unravel a new mechanism whereby Dicer promotes DNA methylation in the nucleus.

The activity of human Dicer has been shown to be regulated by its post-translational modification, such as phosphorylation^25^ and SUMOylation.^26^ During most of oogenesis, phosphorylation of Dicer protein is necessary to trigger Dicer's nuclear translocation in worms, mice and human cells.^27^ Our results demonstrate that most of Dicer proteins in CCA cells had translocated to nucleus in contrast to that seen in the HIBEpic cells (Figure 1b). Further research needs to be done to check whether Dicer translocates to nucleus by its phosphorylation. In addition, we found comparable nuclear expression of Dicer in the LV-saR-Dicer HIBEpic and LV-NC groups (Figure 2c). Dicer which was upregulated in cytoplasm could not translocate to nucleus to regulate DNA methylation in the LV-saR-Dicer HIBEpic cells (Figure 3d). We suspect that in the development of CCA, Dicer is phosphorylated after receiving certain tumor signaling, and translocates to nucleus to regulate DNA methylation. This hypothesis will be verified in our future study.

No clear correlation between Dicer expression and cancer type or disease progression has been reported. Chiosea *et al.*^28^ reported significant changes in Dicer expression had been detected during different stages of lung adenocarcinoma. Some have reported increased Dicer expression in prostate adenocarcinoma cancer^29^ and Burkitt's lymphoma.^30^ In contrast, others have reported reduced Dicer expression in nasopharyngeal carcinoma^31^ and gastric cancer.^32^ In the present study, Dicer expression in CCA cells was significantly higher than that in the HIBEpic cells. There are also many controversies whether Dicer acts as a tumor suppressor^33, 34^ or an oncogene.^35^ In our study, Dicer not only promoted proliferation and invasive properties of CCA cells but also appeared to inhibit apotosis, which is consistent with its role as an oncogene. The discrepancy between the results of various studies may be related to a cell-type-specific effect.

The article "Dicer promotes tumorigenesis by translocating to nucleus to promote SFRP1 promoter methylation in cholangiocarcinoma cells" was published in 2017. Journal: Cell Death Dis.

In conclusion, our study revealed that Dicer translocates to nucleus to promote SFRP1 promoter methylation by coordinating with HP1*α* in CCA cells, and thus promotes CCA progression. The present study broadens our understanding of the complex mechanisms underlying the pathogenesis of CCA and also suggests Dicer as a potential therapeutic target.

## Materials and methods

### Antibodies and tissue samples

The following antibodies were purchased: goat polyclonal anti-HP1*α* (Abcam, Cambridge, MA, USA, ab77256), mouse monoclonal anti-Dicer (Abcam, ab14601), rabbit polyclonal anti-H3K9me3 (Abcam, ab8898), rabbit polyclonal anti-SFRP1 (Abcam, ab4193), mouse monoclonal anti-RNA Polymerase II (Abcam, ab817), rabbit monoclonal anti-cleaved caspase-3 (Cell Signaling Technology, Beverly, MA, USA, no.9664), rabbit monoclonal anti-cleaved PARP (Cell Signaling Technology, no.5625), rabbit polyclonal anti-Dnmt1 (SantaCruz, Dallas, TX, USA, sc-20701), rabbit polyclonal anti-Dnmt3a (SantaCruz, sc-20703), rabbit polyclonal anti-Dnmt3b (SantaCruz, sc-20704), rabbit polyclonal anti-SUV39H1 (Proteintech, Wuhan, China, 10574-1-AP), mouse monoclonal anti-GST (Proteintech, 66001-1-Ig), rabbit polyclonal anti-Histone 3 (Proteintech, 17168-1-AP) and mouse monoclonal anti-*β*-actin (BOSTER, Wuhan, China, BM0626) were used as primary antibody. Normal IgG (Beyotime, Shanghai, China, A7007) was used as a control for co-immunoprecipitation.

Forty human CCA samples and 13 adjacent normal tissues were obtained from the Department of Biliary-Pancreatic Surgery, Tongji Hospital of Huazhong University of Science and Technology (HUST, Hubei, China). Ethics Committee at the Tongji Hospital had approved the study. Written informed consent was obtained from all patients.

### Cell culture and transfection

Human CCA cell lines (Hucct1 and TFK1) and cholangiocyte cell line HIBEpic which were cultured in our laboratory. These were maintained in RPMI 1640 supplemented with 10% fetal bovine serum (FBS) in a humidified incubator containing 5% CO_2_ at 37 °C. While HEK293 cells were cultivated in DMEM/High glucose medium with 10% FBS at 37 °C.

The article "Dicer promotes tumorigenesis by translocating to nucleus to promote SFRP1 promoter methylation in cholangiocarcinoma cells" was published in 2017. Journal: Cell Death Dis.

Small interfering RNA (siRNA) against Dicer gene (Target sequence: 5′-GGAAGAGGCTGACTATGAA-3′), siRNA against SFRP1 gene (Target sequence: 5′-GCCACCACTTCCTCATCAT-3′) and small activating RNA (saRNA) against Dicer gene (Target sequence: 5′-AGCTAAGCTCTCCGGGAAA-3′) were purchased (RiboBio Co., Ltd, Guangzhou, China). The candidates of saRNA were scanned 2 kb upstream of the transcriptional start site of Dicer as previously described.^36^ Transient transfection was performed with Lipofectamine 2000 (Invitrogen, Camarillo, CA, USA) following the manufacturer's instructions. Transfected cells were incubated for 48 h, followed by cell harvesting and analysis.

SaRNA of Dicer lentivirus vector, siRNA of Dicer lentivirus vector and negative control lentivirus (LV-NC, short for LV-siR-negative control) were constructed (Genechem Co., Ltd, Shanghai, China). After extraction from HEK293 cells, the cDNA fragment of target gene was amplified by PCR and then subcloned into the lentiviral vector pGC-LV containing tagged green fluorescent protein (GFP). The final lentiviral construct U6-MCS-Ubi-EGFP was verified by DNA sequencing. The lentiviruses were diluted in 0.3 ml (10^7^ TU/ml) complete medium containing polybrene in 25 ml cell culture flask and incubated at 37 °C for 24 h. Then lentivirus medium was replaced with fresh RPMI1640 medium and the cells were cultured for the next 48 h.

### RNA extraction and quantitative real-time PCR

Total RNA was extracted using Trizol reagent (Invitrogen) as per the manufacturer's protocol. To quantify mRNA, 400 ng of total RNA was synthesized into cDNA using a PrimeScript RT Reagent kit (Takara, Dalian, China). Real-time PCR was performed in a 10 *μ*l reaction mixture with SYBR Premix Ex Taq (Takara) on the iQ5 quantitative PCR detection system (Bio-Rad, Richmond, CA, USA) and the results were analyzed with IQ5 software. The primer sequences for PCR include: Dicer-F:5′-TCACTTCCTGCGGATTTTAGA-3′,Dicer-R:5′-GCTTACCAGGGGACTCGCT-3′SFRP1-F:5′-GAGCCGGTCATGCAGTTCTT-3′,SFRP1-R:5′-CGTTGTCACAGGGAGGACAC-3′.

### Western blot

Protein extracts were subjected to centrifugation at 12 000 × *g* for 15 min at 4 °C. A total of 50 *μ*g of total proteins were separated on 12% polyacrylamide gel and transferred to PVDF membrane (Millipore, Billerica, MA, USA). Protein bands which had been incubated with corresponding antibodies were detected by enhanced chemiluminescence reagents ECL (Millipore).

### GST pull-down

The encoded GST-HP1*α* (GST-Dicer) fusion proteins and the control GST proteins were expressed in BL21 cells. The fusion proteins were arrested by glutathione-Sepharose 4B beads for the GST pull-down assays, and HEK293 cells extracts were added. Binding was performed for 3 h under rotation at 4 °C and the beads were washed with ice-cold PBS. The supernatant was loaded to gels followed by western blot identification using anti-Dicer (or anti-HP1*α*).

The article "Dicer promotes tumorigenesis by translocating to nucleus to promote SFRP1 promoter methylation in cholangiocarcinoma cells" was published in 2017. Journal: Cell Death Dis.

### Co-immunoprecipitation

Co-immunoprecipitation of HP1*α*-associated proteins was performed using 2.5 *μ*g anti-HP1*α* antibodies and 20 *μ*l Protein A+G Agarose beads (Beyotime) according to manufacturer's instructions. Each immunoprecipitated protein was detected by western blot analysis using antibodies such as anti-Dicer, anti-Dnmt1, anti-Dnmt3a, anti-Dnmt3b, anti-SUV39H1 and anti-H3K9me3. IgG was used as a control for co-immunoprecipitation.

### Immunohistochemistry

Forty CCA tissue specimens and 13 adjacent normal tissue specimens were deparaffinized, rehydrated through graded alcohol, washed with Tris-buffered saline (TBS), and processed using a streptavidin-biotin-peroxidase complex method. Antigen retrieval was performed by autoclaving the slides in 10 mM citric acid buffer. Samples were incubated overnight with 1:500 diluted anti-Dicer antibodies at 4 °C. The corresponding secondary antibody was used for 30 min at 37 °C. Samples were counterstained with hematoxylin before dehydration and mounting. Nuclei which were stained blue with hematoxylin, and cytoplasm were scored for Dicer expression, respectively.

Semi-quantitative scoring of immunohistochemical staining was performed using percentage of stained cells (0: <5% positive cells; 1: 5% to 24% positive cells; 2: 25% to 49% positive cells; 3: 50% to 74% positive cells and 4:≥75% positive cells) and intensity of positive staining (0: absence of staining; 1: weak; 2: moderate; 3: strong staining). Stain scoring=intensity × positive rate (absent, 0–1; mild, 2–4; moderate, 5–8; and strong, 9–12).

### Chromatin immunoprecipitation (ChIP)

Approximately 10^7^ cells were fixed with 1% formaldehyde to crosslink endogenous proteins and DNA. Samples of sonicated chromatin were immunoprecipitated with primary antibodies and protein A+G Agarose beads. IgG served as a negative control. Immunoprecipitated DNA and input DNA were analyzed by quantitative real-time PCR using specific primers:

SFRP1-F:5′-GGTTGCAGTCAGCGGAGATA-3′,SFRP1-R:5′-GGAGCCTGGATCATACTTGC-3′Actin-F:5′-CCCTCCTCCTCTTCCTCAATCT-3′,Actin-R:5′-AACGGCGCACGCTGATT-3′.

### Bisulfite sequencing PCR (BSP)

BSP primers were designed according to online MethPrimer program (http://www.urogene.org/methprimer). Primer sequences for BSP were as following: BSP-SFRP1-F:5′-TYGGGAGTTGATTGGTTG-3′, BSP-SFRP1-R:5′-CTTCCAAAAACCTCCRAAAA-3′. BSP reactions were performed using ddH_2_O, 10 × PCR buffer, dNTP mix, PCR primer, rTaq and bisulfite converted DNA samples in 25 *μ*l final volume. The PCR product was subcloned into pMD19-T vector, and 10 clones from each group were randomly selected and sent for Sanger sequenced by Oebiotech Co (Shanghai, China).

The article "Dicer promotes tumorigenesis by translocating to nucleus to promote SFRP1 promoter methylation in cholangiocarcinoma cells" was published in 2017. Journal: Cell Death Dis.

### Flow cytometry

Cells were trypsinized and centrifuged at 1000 r.p.m. for 5 min, washed, and resuspended with cold PBS for three times. Then they were fixed with 70% ethanol at −20 °C for 24 h, followed by washing, centrifugation in 500 *μ*l PBS. The cells were stained with 300 *μ*L PI (0.05 mg/ml) for another 30 min in the dark. The fluorescence of PI was measured by flow cytometer (Becton Dickinson Franklin Lakes, NJ, USA). Cell proliferation status was evaluated mainly by the ratio of S-phase.

### Cell proliferation assay

Cells were seeded at a density of 5 × 10^3^ cells per well in a 96-well plate containing 100 *μ*l RPMI 1640 medium and 10% FBS. Cell Counting Kit-8 (CCK-8) (Dojindo, Tokyo, Japan) reagent was added at 48 h after seeding and incubated at 37 °C for 1 h. The optical density (OD) at 450 nm was measured by a microplate reader (Bio-Rad).

### Cell migration and invasion assay

CCA cells were seeded in 24-well plates and the confluent monolayer cells (at 90% confluence) were scratched with a sterile 100-*μ*l pipette tip. Images of the migrated cells were taken using a digital camera (Leica, Heerburg, Germany) at 0 and 24 h after scratching. The extent of wound healing was assessed by the distance of migration into the denuded area. For invasion assay, upper chamber filters of the transwell were coated with Matrigel mixed with serum-free medium (diluted at 1:8) (BD Biosciences, San Jose, CA, USA) according to the manufacturer's instructions. After 36 h, cells that did not migrate or invade were removed using a cotton swab. Invasive cells at the bottom of the membrane were fixed in 4% paraformaldehyde, stained with 1% crystal violet and counted under a microscope.

### Tumorigenicity assay in nude mice

2 × 10^5^ Hucct1 cells in 200 *μ*l PBS were subcutaneously injected into four-week-old male BALB/C nude mice, purchased from the Beijing HFK Bioscience Co., Ltd, Beijing, China. Tumor growth was measured with calipers every 4 days and the tumor volumes were calculated using the formula: 0.5 × length × width^2^. All mice were killed after 4 weeks. The study was approved by the Experimental Animal Ethics Committee at the Tongji Medical College of Huazhong University of Science and Technology.

### Illumina 450 K methylation microarray

The Human Methylation 450 K microarray evaluates 450 000 methylation sites across the genome, which covers 96% of all CpG islands. The chip is used to evaluate the average DNA methylation rate (AVG_Beta) of genomic regions. When Delta_Beta [Delta_Beta=case(AVG_Beta)−control(AVG_Beta)] is >0.17 or <−0.17, the gene is defined as the differentially methylated gene.

The article "Dicer promotes tumorigenesis by translocating to nucleus to promote SFRP1 promoter methylation in cholangiocarcinoma cells" was published in 2017. Journal: Cell Death Dis.

After bisulfite treatment, the whole genome was amplified, enzymatically fragmented and hybridized to the 450 K Illumina Infinium Methylation BeadChip kits (Illumina, Inc., San Diego, CA, USA). Allele-specific single-base extension and staining were performed and the BeadChips imaged on Illumina BeadArray Reader. The image intensity was extracted using Illumina's BeadScan software (Illumina iScan scanner). Array data export processing and analysis were performed using Illumina GenomeStudio v2011.1 (Methylation Module v1.9.0) and the statistical computing package R 3.0.2. Data analyses including differential methylation analysis, gene ontology analysis and pathway analysis were performed.

### Statistical analysis

All data were representative of three independent experiments and were presented as the mean±S.D. A two-sample *t*-test was performed to analyze two independent samples, whereas analysis of variance was conducted for comparison among groups. GraphPad Prism 5.0 (GraphPad Prism Software Inc., San Diego, CA, USA) was used to calculate *P*-values; *P*<0.05 was considered statistically significant.

## Figures and Tables

**Figure 1:** Dicer is upregulated and translocates to nucleus to form complex with HP1*α* in CCA cells. (**a**) IHC analysis of Dicer expression in 40 CCA tissue samples and 13 pericancerous normal tissues. Representative images (left) and independent samples *t*-test analysis of Dicer scoring (right) are shown. Scale bar, 25 *μ*m (red line). (**b**) Western blot analysis of Dicer in Hucct1, TFK1 and HIBEpic cell lines. Actin and Histone 3 was used as internal control for cytoplasm and nucleus, respectively. (**c**) The interaction of HP1*α* with Dicer was determined by GST pull-down treated with RNase A in HEK293 cells. (**d**) Co-immunoprecipitation of Dicer (or HP1*α*) protein from Hucct1 and HIBEpic cells with anti-HP1*α* (or anti-Dicer) antibodies, followed by western blot. (**e**) Co-immunoprecipitation of Hucct1 cells with anti-HP1*α* antibodies, followed by western blot. *P<0.05

**Figure 2:** Dicer regulates chromatin modifications in CCA cells. (**a**) Levels of Dicer mRNA in Hucct1, TFK1 and HIBEpic cells following transfection with lentiviral vectors. Actin was used as an internal control. Protein levels of Dicer in cytoplasm (**b**) and nucleus (**c**) following transfection with lentiviral vectors. Actin and Histone 3 were used as loading controls. (**d**) Protein levels of H3K9me3 in Hucct1, TFK1 and HIBEpic cells were detected by western blotting. Histone 3 was used as a loading control. The relative gray values of H3K9me3 above each lane were normalized against Histone 3. (**e**) Human Methylation 450K analysis of the changed DNA methylation patterns between LV-siR-Dicer and LV-NC Hucct1 cells. **P<0.01

**Figure 3:** Dicer promotes SFRP1 promoter methylation and its expression negatively correlated with that of SFRP1 in the CCA samples. (**a**) Listing of average DNA methylation rate of eight most differentially methylated genes between LV-siR-Dicer and LV-NC, including four hypermethylated genes and four hypomethylated genes. (**b**) Graphic model of the CpG islands of SFRP1 promoter and primer amplification products of ChIP and BSP assays. (**c**) Indicated cells were subjected to ChIP assays for Dicer, HP1*α* and H3K9me3 enrichment of SFRP1 promoter and Actin promoter. IgG served as a negative control. Relative enrichment fold=[%(ChIP/Input)]/[%(IgG/Input)]. Enrichment fold of RNA Polymerase II in the housekeeping gene Actin promoter served as positive control for the ChIP assays. (**d**) Indicated cells were subjected to BSP assays. Each row represents a single sequence, and the dots represent the CpG sites. Gray and black dots represented unmethylated and methylated CpGs, respectively. (**e**) Levels of SFRP1 mRNA in CCA cells were detected by qRT-PCR among LV-siR-Dicer, LV-NC and LV-NC+5-aza-dC groups. Actin was used as an internal control. (**f**) The mRNA expression of SFRP1 showed a negative correlation with that of Dicer in the 40 CCA tissue specimens. Statistical analysis was performed using Pearson's correlation coefficient. (r=−0.47, *P*<0.01). *P<0.05, **P<0.01

**Figure 4:** Dicer promotes proliferation and invasion by silencing SFRP1 expression, inhibits apoptosis of CCA cells and associates with clinicopathology. (**a**) Protein levels of SFRP1 detected on western blotting in indicated CCA cells. Actin was used as a loading control. (**b**) Flow cytometric analysis of cell cycle distribution. Cell proliferation status was assessed mainly by the ratio of S-phase cells. (**c**) Indicated CCA cells were subjected to CCK-8 assay for 4 days. (**d**) Indicated cells were subjected to wound healing assays to assess migration. Representative images (left) and statistical comparison of the indicated groups (right) were shown. (**e**) Indicated cells were subjected to Transwell assays for invasion. (Magnifications: × 200). (f) Protein expression of cleaved caspase-3 and PARP reflecting status of apoptosis in the indicated CCA cells. (**g**) Representative photographs of tumors in nude mice (*N*=6 per group) derived from LV-siR-Dicer and LV-NC Hucct1 cells. Statistical analysis of tumor volume every 4 days are shown in the under panel. (**h**) Results of qRT-PCR showing mRNA expressions of SFRP1 and Dicer mRNA in tumor tissues from nude mice. Actin was used as an internal control. (**i**) Kaplan–Meier overall survival curves for nine patients with low Dicer expression and 31 patients with high Dicer expression. *P<0.05, **P<0.01

**Figure 5:** Schematic illustration of the role of Dicer in CCA investigated in the present study. With the progression of CCA, Dicer translocates from the cytoplasm to nucleus after receiving certain signaling, and interacts with HP1*α*. The Dicer/HP1*α* complex recruits SUV39H1 to trimethylate H3K9 and Dnmts to methylate SFRP1 promoter, which represses transcription

**Table 1:** Association between Dicer expression in 40 CCA tissue specimens and clinicopathological characteristics

**Characteristics**	**Number of patients**	**Low expression (IHC staining index:≤6)**	**High expression (IHC staining index:>6)**	***P*-value**
*Age (years)*				
≤60	14	5	9	0.23
>60	26	4	22	
				
*Sex*				
male	27	6	21	1.00
female	13	3	10	
				
*Tumor size (cm)*				
≤3	19	8	12	0.02^a^
>3	21	1	19	
				
*Pathology grade*				
Low (I+II)	26	8	18	0.12
High (III+IV)	14	1	13	
				
*Lymph node metastasis*				
Negative	17	7	10	0.02^a^
Positive	23	2	21	

Abbreviations: CCA, cholangiocarcinoma; IHC, immunohistochemistry

a Significant correlation
